# Fibril specific, conformation dependent antibodies recognize a generic epitope common to amyloid fibrils and fibrillar oligomers that is absent in prefibrillar oligomers

**DOI:** 10.1186/1750-1326-2-18

**Published:** 2007-09-26

**Authors:** Rakez Kayed, Elizabeth Head, Floyd Sarsoza, Tommy Saing, Carl W Cotman, Mihaela Necula, Lawrence Margol, Jessica Wu, Leonid Breydo, Jennifer L Thompson, Suhail Rasool, Tatyana Gurlo, Peter Butler, Charles G Glabe

**Affiliations:** 1 Department of Molecular Biology and Biochemistry, University of California, Irvine, CA 92697, USA; 2 Department of Neurology and Institute for Brain Aging & Dementia, University of California, Irvine, CA 92697, USA; 3 Larry Hillblom Islet Research Center, David Geffen School of Medicine, University of California, Los Angeles, CA 90095-7073, USA

## Abstract

**Background:**

Amyloid-related degenerative diseases are associated with the accumulation of misfolded proteins as amyloid fibrils in tissue. In Alzheimer disease (AD), amyloid accumulates in several distinct types of insoluble plaque deposits, intracellular Aβ and as soluble oligomers and the relationships between these deposits and their pathological significance remains unclear. Conformation dependent antibodies have been reported that specifically recognize distinct assembly states of amyloids, including prefibrillar oligomers and fibrils.

**Results:**

We immunized rabbits with a morphologically homogeneous population of Aβ42 fibrils. The resulting immune serum (OC) specifically recognizes fibrils, but not random coil monomer or prefibrillar oligomers, indicating fibrils display a distinct conformation dependent epitope that is absent in prefibrillar oligomers. The fibril epitope is also displayed by fibrils of other types of amyloids, indicating that the epitope is a generic feature of the polypeptide backbone. The fibril specific antibody also recognizes 100,000 × G soluble fibrillar oligomers ranging in size from dimer to greater than 250 kDa on western blots. The fibrillar oligomers recognized by OC are immunologically distinct from prefibrillar oligomers recognized by A11, even though their sizes overlap broadly, indicating that size is not a reliable indicator of oligomer conformation. The immune response to prefibrillar oligomers and fibrils is not sequence specific and antisera of the same specificity are produced in response to immunization with islet amyloid polypeptide prefibrillar oligomer mimics and fibrils. The fibril specific antibodies stain all types of amyloid deposits in human AD brain. Diffuse amyloid deposits stain intensely with anti-fibril antibody although they are thioflavin S negative, suggesting that they are indeed fibrillar in conformation. OC also stains islet amyloid deposits in transgenic mouse models of type II diabetes, demonstrating its generic specificity for amyloid fibrils.

**Conclusion:**

Since the fibril specific antibodies are conformation dependent, sequence-independent, and recognize epitopes that are distinct from those present in prefibrillar oligomers, they may have broad utility for detecting and characterizing the accumulation of amyloid fibrils and fibrillar type oligomers in degenerative diseases.

## Background

The accumulation of misfolded proteins and peptides as amyloid deposits is a characteristic feature of many degenerative diseases, such as Alzheimer disease (AD), although the pathological significance of these deposits remains unclear. In AD, several different types of deposits containing the amyloid Aβ peptide have been recognized, including dense cored, neuritic, diffuse and "cotton wool" plaques [1-3]. Sites of intracellular accumulation of Aβ have also been identified [4-8]. The relationships and pathological significance of these accumulated deposits remain a matter of debate. The pathological significance of the fibrillar plaques is a matter of debate, since cognitively normal aged individuals frequently have large amounts of fibrillar deposits [9,10] and soluble oligomeric forms of Aβ correlate better with dementia [11,12]. It has also been suggested that the large insoluble amyloid deposits may serve as reservoirs that release toxic soluble oligomers [13]. It is widely accepted that diffuse amyloid deposits are "non-fibrillar" based on a lack of binding of fibril-specific dyes, like Congo red (CR) and ThioS. Senile plaques and "cored" plaques stain with CR and ThioS, while most diffuse plaques are negative [9]. Thioflavin dyes have served as the basis for the development of contrast agents to image amyloid accumulation in vivo in humans, although these dyes do not label diffuse plaques in human AD brain nor the amyloid deposits that accumulate in transgenic mouse models of AD.

Plaques have also been characterized immunologically. Monoclonal antibodies specific for the carboxyl terminus of Aβ indicate that diffuse plaques primarily contain Aβn-42, while dense core and neuritic plaques contain both Aβn-40 and Aβn-42 [14,15]. More recently, conformation-dependent antibodies have been reported that recognize a generic epitope that is specific to many types of amyloid fibrils and not soluble monomer regardless of their sequences [16,17]. The WO1 antibody has been reported to bind to a generic fibril epitope [17], but this antibody also recognizes morphologically distinct "protofibrils" [18]. Whether this epitope recognized by WO1 is specific to the fibrillar state or is also displayed on prefibrillar aggregates or oligomers has yet to be determined. Other conformation dependent antibodies (A11) have been reported that specifically recognize a generic epitope common to prefibrillar oligomers and not fibrils, monomers or natively folded precursor proteins [19]. These oligomers are widely believed to represent a primary toxic or pathological species and are called "prefibrillar" because they kinetically precede fibril formation and disappear after fibrils have formed [20,21]. While A11 stains small focal or punctuate deposits in AD tissue, it does not stain diffuse plaques or other plaque types, indicating that diffuse deposits are not accumulations of prefibrillar oligomers.

Here we report a conformation dependent, fibril specific polyclonal antisera that recognizes a generic epitope that is associated with amyloid fibrils and soluble fibrillar oligomers that is distinct from prefibrillar oligomers. Like other conformation dependent antibodies, it does not recognize natively folded APP or monomer. This antibody may have considerable utility for localizing and quantitating fibril related aggregates in tissues and biological fluids.

## Results

### Fibril specificity of OC antisera

The specificity of OC antisera was examined by ELISA and dot blot analysis of monomeric, prefibrillar oligomeric and fibrillar Aβ and other types of amyloids (Fig. 1). ELISA analysis indicates that OC is conformation dependent and fibril specific because it recognizes Aβ fibrils, but not Aβ prefibrillar oligomers or Aβ monomer (Fig. 1A). OC recognizes a generic epitope that is associated with the fibrillar amyloid state regardless of the sequence because it reacts equally well with α-synuclein fibrils and islet amyloid polypeptide (IAPP) fibrils. Dot blot analysis confirms that the fibril epitope of both Aβ and poly Q (Q36) fibrils is recognized by OC and is complementary and mutually exclusive with the generic prefibrillar epitope of both Aβ and polyQ oligomers that is recognized by A11. A11 does not recognize the fibrillar samples that stain with OC, while OC does not stain the prefibrillar samples recognized by A11 (Fig. 1B). The size distribution of Aβ aggregates that are recognized by OC and A11 was determined by western blotting of fibrillar and prefibrillar oligomer Aβ samples (Fig. 2). Aβ42 fibrils contain 6E10 and 4G8 reactive bands at the positions of 4.5 kDa monomer, dimer, tetramer and a broad smear of aggregates up to the top of the gel. Prefibrillar oligomer Aβ42 samples contain A11 positive aggregates of the same approximate size range as fibrils that are stained by 4G8, but the prefibrillar oligomers are not stained by 6E10. We have previously reported that 6E10 does not stain prefibrillar oligomers prepared by dilution of a stock solution of Aβ42 in 100 mM NaOH in PBS, but it does recognize prefibrillar oligomers formed in water at pH 2.5 and 6E10 recognizes random coil monomer and amyloid fibrils [22]. These results indicate that prefibrillar Aβ oligomers are polymorphic at the 6E10 epitope and that the Aβ monomer in the prefibrillar oligomer preparation has a stable conformation that is not reactive with 6E10. OC anti-fibril antiserum stains the Aβ42 dimer band and higher aggregates from fibrillar samples, but does not stain Aβ monomer (Fig. 2). However, OC does not stain the prefibrillar oligomer aggregates that are stained by A11. A11 stains bands corresponding to tetramer and a broad distribution of aggregates centred on a molecular weight of approximately 60 kDa, indicating that fibrillar oligomers are conformationally distinct from prefibrillar oligomers even though their sizes are broadly overlapping. The size of the bands detected by OC and A11 depend on the time of aggregation with the size increasing with incubation time (data not shown).

**Figure 1:** **Characterization of OC antiserum**. A. ELISA analysis. Plates were coated with homogenous samples of Aβ fibrils, Aβ monomer, Aβ prefibrillar oligomers, and α-synuclein and IAPP fibrils. The samples were reacted with OC serum which indicates that all types of fibrils and not Aβ monomer or prefibrillar oligomers react with OC. B. Dot blot analysis of Aβ42 and polyQ36 prefibrillar oligomers and fibrils. Aβ42 and polyQ fibrils only stain with OC serum, while Aβ42 and polyQ prefibrillar oligomers only react with A11.

**Figure 2:** **Western blot analysis of Aβ42 fibrils and prefibrillar oligomers**. Aβ42 fibrils (F) and prefibrillar oligomers (O) were run on SDS polyacrylamide gels, transferred to nitrocellulose and probed with 6E10, 4G8, OC and A11 antibodies as indicated at the top of the panel. Both fibrillar and prefibrillar oligomer samples contain bands that react with 4G8 ranging from monomer up to the size of material that accumulates at the top of the gel. OC only stains the bands from fibrillar samples of approximately dimer and above. A11 only stains the prefibrillar oligomer samples. 6E10 does not stain prefibrillar Aβ oligomer samples formed at pH 7.4 as previously reported [22].

### Characterization of soluble fibrillar oligomers

The fact that low MW species are recognized on western blots by the OC anti fibril antibody, which are conformationally distinct from the prefibrillar oligomers that react with A11, suggests that at least two distinct types of oligomers exist: fibrillar oligomers and prefibrillar oligomers. We characterized the solubility and size distribution of OC positive oligomers under non-denaturing conditions by ultracentrifugation and size exclusion chromatography. Both fibril preparations prepared in HFIP/water [19] and ADDL preparations prepared in DMSO and cold F12 medium [23] contain a substantial amount of OC positive 100,000 × G soluble material, suggesting that they contain fibrillar oligomers (Fig. 3A). Samples prepared by dilution of DMSO stock solutions of Aβ42 were also fractionated by size exclusion chromatography and the resulting fractions probed with OC. The results indicate that a broad distribution of oligomer sizes from approximately 8 kDa to 200 kDa is recognized by OC (Fig. 3B). These results are consistent with the sizes identified by western blots (Fig. 2). The data suggest that these fibrillar oligomers have Aβ peptides arranged in the same conformation as in fibrils suggesting that they may represent small pieces of fibrils or fibril nuclei.

**Figure 3:** **Solubility and size distribution of fibrillar Aβ42 oligomers under physiological conditions**. **A**. Aβ42 aggregates were prepared in HFIP-H20 and DMSO-F12 medium as described in Materials and Methods and centrifuged at 100,000 × G for 1 hr. The supernatant and pellet fractions were separated and the pellet resuspended in an equal volume of PBS. Aliquots of the supernatant and pellet were dotted on nitrocellulose and probed with OC antisera. Both the soluble and insoluble fractions contain significant amounts of OC reactive material. B. Aβ42 aggregates formed in DMSO were fractionated by size exclusion chromatography on a Toso-Haas 2000 SWXL column, 1 minute fractions collected and dotted on nitrocellulose and probed with OC antisera. The elution profile detected by UV absorbance is shown in the top panel. The bottom panel shows the OC immunoreactivity which is detected in fractions from 8–14 minutes, indicating that low MW Aβ oligomers are immunoreactive with OC. The arrows indicate the positions of the void volume (Vo), included volume (Vi) and the elution positions of molecular weight standards.

### Conformation dependent immune response is independent of antigen sequence

Since both A11 and OC recognize generic epitopes that do not depend on a particular amino acid sequence, we tested whether the immune response to other types of prefibrillar oligomers and fibrils is also specific for generic conformation dependent epitopes. We synthesized an oligomer mimic of islet amyloid polypeptide (IAPP) by coupling IAPP carboxy-terminal thioester to colloidal gold particles as previously described [19]. We used IAPP oligomer mimics and IAPP fibrils to immunize rabbits and we characterized the specificity of the immune response by dot blot. Immunization of rabbits with IAPP oligomer mimics gives rise to a prefibrillar oligomer-specific immune response that is indistinguishable from that obtained with Aβ prefibrillar oligomer mimics (Fig. 4). We call this serum I11 to indicate its derivation from IAPP antigen and its similarity to A11. Like A11, I11 recognizes prefibrillar oligomers derived from Aβ, α-synuclein and IAPP, but not monomers or fibrils on dot blots (Fig. 4A). Western blots of prefibrillar oligomer samples probed with I11 give the same staining pattern as A11 (Fig. 4B). Similarly, rabbits vaccinated with IAPP fibrils give rise to a fibril specific immune response that recognizes Aβ fibrils and does not recognize monomer or prefibrillar oligomers (Fig. 5). The resulting serum is called LOC (Like OC). Taken together these results demonstrate that the immune response to oligomer mimics and fibrils is predominantly conformation dependent and sequence independent.

**Figure 4:** **Comparison of A11 and I11 antibody specificity**. A. Dot blots. Aβ monomer, Aβ prefibrillar oligomers (prepared in HFIP-H20, pH 2.5), Aβ fibrils and α-synuclein and IAPP prefibrillar oligomers were spotted on nitrocellulose strips and probed with A11, I11 and 6E10 as a control. A11 and I11 antibodies demonstrate the same specificity for prefibrillar oligomers and do not react with monomer or fibrils. 6E10 stains the Aβ-containing samples, including prefibrillar oligomers formed at acid pH. B. Western blots. Prefibrillar oligomer samples of calcitonin (Lane 1), insulin (Lane 2) and prion peptide 106–126 (Lane 3) were probed with A11 and I11, which give the same staining pattern.

**Figure 5:** **Comparison of LOC and OC antisera specificity**. Aβ monomer, prefibrillar oligomers and fibrils were spotted on nitrocellulose strips and probed with LOC and OC antisera. Both LOC and OC react only with fibrillar samples.

### OC and LOC immunoreactivity in human AD tissue

We also investigated the distribution of OC and LOC staining in human AD brain using two AD cases with Aβ and NFT pathology. Figure 6 shows significant OC immunolabeling in the hippocampus and temporal cortex. All types of Aβ deposits stain with OC, including diffuse, neuritic and cored plaques (Fig. 6) and cerebrovascular amyloid deposits (data not shown). Therefore, OC staining of diffuse amyloid deposits indicates that they share the fibrillar immunological structure of other amyloid deposits even though they do not stain with "fibril specific" dyes, such as thioflavin S. Intracellular NFTs do not stain with OC, even though it has been suggested that they contain local β-sheet character [24]. Immunolabeling was virtually abolished when the antibody was incubated with a 100-fold concentration of the fibrillar antigen prior to incubation with the tissue (Fig. 6E, F). We next compared OC and LOC immunoreactivity by confocal microscopy as both antibodies recognize similar assembly states of Aβ. The staining patterns of the two antibodies overlap significantly within plaques of an AD case since most of the fluorescent signals are coincident in the merged image (Fig. 6G–I). Since LOC is raised against IAPP, this indicates that the plaque staining is conformation dependent and not due to a small amount of linear Aβ sequence specific antibodies that may contaminate OC.

**Figure 6:** **Immunolabeling characteristics of OC in an AD case and preabsorption controls**. Extensive OC labeling was observed in the hippocampus (A), subiculum (B) and frontal cortex (C) in AD. A higher magnification photograph illustrates that OC positive deposits were dense and consisted of fine fibrillar material (D). Preabsorption with a 100-fold concentration of OC antigen leads to a significant reduction in immunolabeling in the frontal cortex (E &F). Significant overlap was observed between OC positive immunoreactivity (Red – G) and LOC positive immunoreactivity (Green-H) suggesting that the two antibodies recognize similar deposits (Overlap is yellow – I). Magnification in A, B, C – 1.25×, D – 20×, E, F – 4× and G, H, I – 40×.

Lysates of human AD brain were also analyzed biochemically with OC. OC immunoreactivity was found in the Triton X-100 100,000 × G insoluble fraction of all AD patients examined (Fig. 7). This appeared as very high MW material that sticks at the top of the gel or in the stacking gel after boiling in SDS sample buffer. After stripping and reprobing, this high MW material also stains with 4G8 (anti-Aβ17–28) antibody. No OC staining was observed in the Triton X-100 soluble fraction, indicating that OC does not recognize APP and that the level of fibrillar oligomers in this fraction is below the limit of detection by this method (data not shown). The insoluble fraction was also dissolved in formic acid and dried prior to SDS gel electrophoresis. After formic acid treatment, OC staining is abolished although 4G8 staining is retained after stripping and reprobing, indicating that the staining is conformation dependent. The 4G8 staining reveals that formic acid treatment has a small effect on breaking down the high MW material with more immunoreactivity at the top of the running gel and a small amount of low MW Aβ immunoreactivity. Interestingly, the OC immunoreactivity is insensitive to formic acid treatment, typically used to enhance Aβ immunostaining, after fixation of human AD brain tissue with paraformaldehyde. The immunoreactivity is insensitive to pretreatment of sections with up to 90% formic acid (data not shown).

**Figure 7:** **Western blot analysis of Triton X-100 insoluble fractions from human AD brain lysates**. Frontal cortex samples, either untreated or formic acid treated, from 6 individual AD brains were dissolved in SDS sample buffer and electrophoresed on polyacrylamide gels and probed with OC or 4G8 as a control. Upper panels: For untreated samples, both OC and 4G8 detect high molecular weight material that accumulates at the top of the gel. Bottom panels: After formic acid treatment, 4G8 detects some lower MW bands in addition to formic acid resistant high MW material, while the staining by OC is abolished, indicating that the staining is conformation dependent.

### OC staining of islet amyloid deposits

The broad specificity of OC for different types of amyloid fibrils suggests that it may have broad utility in staining different types of amyloid deposits. We also examined the OC staining of islet amyloid deposits in the pancreas of human IAPP transgenic mouse model of type II diabetes [25]. OC stains intra and extracellular IAPP amyloid deposits, indicating that the IAPP deposits display the same fibril related generic epitope in vivo that they display in vitro (Fig. 8). Together, these results indicate that the broad fibril specific immunoreactivity of OC may be useful for identifying a number of different types of amyloid deposits in human disease.

**Figure 8:** **OC staining of pancreatic section from Tg mouse model of type II diabetes expressing human IAPP (obese hemizygous human IAPP transgenic mouse)**. OC labeling (red) was detected within the islets in insulin-positive (green) beta cells and in the extracellular amyloid deposits.

## Discussion

Amyloidogenic proteins and peptides can adopt a number of distinct assembly states and a key issue is which of these assembly states are more closely associated with pathogenesis. Conformation dependent antibodies that specifically recognize these distinct assembly states offer the potential of providing insight into which distinct assembly states accumulate in disease and are pathologically significant. We have prepared polyclonal antisera that recognize a generic epitope specific to amyloid fibrils. These antibodies are similar to other fibril specific antibodies that have been previously reported [16,17]. One of the major insights we have gained from examining the properties of OC polyclonal antiserum and comparing it to A11, is that there are at least two distinct types of amyloid oligomers: prefibrillar oligomers and fibrillar oligomers. The idea of fibrillar oligomers may seem counter intuitive because fibrils are often thought of as large insoluble structures, but the fact that OC recognizes small soluble oligomers in the range of dimers to 250 kDa that are not recognized by A11 indicates that these oligomeric species are conformationally related to fibrils and conformationally distinct from prefibrillar oligomers. It is not surprising that small fibrillar oligomers or pieces of fibrils exist, because it is known that fibril assembly is a nucleation-dependent process and these soluble fibrillar oligomers may represent fibril nuclei or seeds.

The fact that the epitopes recognized by OC and A11 are generic and mutually exclusive indicate that the conformational difference between fibrils and prefibrillar oligomers is a widespread and fundamental distinction for many different types of amyloids. This fundamental conformational difference forms an ideal and rational basis for the nomenclature of amyloid assembly states. We propose that oligomers can be classified as at least two distinct types: prefibrillar oligomers and fibrillar oligomers (Fig. 9). Prefibrillar oligomers are defined as an assembly state that can ultimately convert to a fibrillar state by concerted or "en bloc" conformational conversion, while fibrillar oligomers grow predominantly by addition of monomer to the ends without undergoing further conformational change. This elongation would involve a conformation conversion at the level of the monomer. The distinction between a fibrillar oligomer and a fibril is on the basis of size and it seems likely that there is a continuous distribution of potential sizes that vary by a single monomeric subunit. There is no obvious demarcation between fibrillar oligomers and fibrils, suggesting that the distinction is necessarily arbitrary and operational. This does not imply that size is not important pathologically as small oligomers may have more diffusional freedom than large fibrils and therefore may be able to move more freely and bind reversibly to cellular targets.

**Figure 9:** **Schematic representation of the distinct types of amyloid oligomers and their relationships to amyloid fibrils**. Amyloid aggregation pathways begin with misfolded amyloidogenic monomer (top) and can diverge in two directions depending on which conformation it adopts. It can aggregate to form prefibrillar oligomers by adopting the conformation recognized by A11 (left pathway). These prefibrillar oligomers then align to form protofibrils (not shown) and undergo another conformation change "en bloc" to form fibrils. They are termed prefibrillar oligomers because they are transient intermediates that ultimately become fibrils. Alternatively, amyloidogenic monomer can aggregate to adopt a fibrillar conformation recognized by OC antibody (right pathway). The resulting fibrillar oligomers may represent fibril nuclei which are the minimal stable aggregate that is capable of elongating by recruiting additional monomers. Addition of monomers on to the ends of fibrillar oligomers and fibrils result in fibril growth. The distinction between fibrillar oligomers and fibrils is based on an arbitrary size difference as no conformation difference is apparent. Fibrils may be distinct from fibrillar oligomers on the basis of their content of multiple protofilaments (not shown) but this does not necessarily imply a necessary conformation difference in their integral peptide constituents.

The size of amyloid oligomers is not a reliable indicator of their conformation or aggregation state. Prefibrillar oligomers and fibrillar oligomers display broadly overlapping size distributions, yet they are conformationally distinct by virtue of the fact that they display mutually exclusive epitopes. Since soluble amyloid oligomers are widely believed to represent the primary pathological species rather than insoluble amyloid fibrils, this raises the question of which type of oligomer is important for pathogenesis and whether prefibrillar and fibrillar oligomers have distinct pathogenic mechanisms. Prefibrillar oligomers have been reported in human AD brain [19]. It is not yet clear whether fibrillar oligomer exist in human AD brain and whether this correlates with pathology, but this is the subject of further studies. Our results also suggest that a lack of staining with thioflavin dyes and Congo red may not be a reliable indicator of non-fibrillar conformation. These dyes do not stain diffuse amyloid deposits although all amyloid deposits including diffuse plaques stain with OC, indicating that they display the fibril-specific epitope. It has been suggested that insoluble amyloid plaques may represent a reservoir for soluble oligomer production. If so, our data would suggest that this would be a source of fibrillar oligomers rather than prefibrillar oligomers, since all types of amyloid plaque deposits stain intensely with OC.

Recent evidence indicates that prefibrillar oligomers are not an obligate intermediate for amyloid fibril formation and that they represent alternative aggregation pathways and in vitro. Fibrils form under conditions that do not support the formation of prefibrillar oligomers and drugs that inhibit prefibrillar oligomer formation have no effect on fibril formation or they actually promote fibril formation [22,26]. If prefibrillar oligomers are not obligate intermediates for fibril formation *in vivo*, this would suggest that amyloid fibrils could deposit without forming prefibrillar oligomers. If prefibrillar oligomers are the primary toxic species, the direct formation of fibrils in the absence of prefibrillar oligomers could explain why some cognitively normal individuals have large amounts of insoluble amyloid fibrils.

We also investigated whether the conformation dependent immune response that gives rise to antibodies that recognize generic epitopes associated with distinct aggregations states is independent of the peptide sequence used as an antigen. We immunized rabbits with oligomer mimics and amyloid fibrils derived from the islet amyloid polypeptide and compared the specificity of the immune response to antibodies elicited in response to Aβ derived oligomer mimics and amyloid fibrils. We found that the resulting immune sera are functionally equivalent with the islet oligomer mimic antiserum, I11, recognizing the same prefibrillar oligomers as A11 and the islet fibril antibodies, LOC recognizing the same fibrillar epitope as OC. This suggests that the immune response to amyloid aggregates is predominantly conformation dependent, rather than sequence specific. This observation may have some practical utility. The staining of Aβ amyloid plaques with LOC rules out the possibility that the plaque staining is due to residual Aβ sequence specific immunoreactivity. It also suggests the possibility that oligomers and fibrils may be specifically targeted by vaccination with non-human amyloid sequences that could give rise to a therapeutic immune response while avoiding potential autoimmune complications.

## Conclusion

Fibrils and fibrillar amyloid oligomers display a unique generic epitope that is distinct from the generic epitope displayed by prefibrillar oligomers. Conformation dependent antibodies specific for these generic epitopes may have broad utility for specifically targeting these distinct aggregation states in amyloid related degenerative diseases.

## Methods

### Antigen and antibody preparation

Fibril antigens were prepared by stirring 2 mg/ml Aβ42 peptide in 50% HFIP/H2O, 0.02% sodium azide for 7 days. Afterwards, the HFIP was evaporated under a stream of nitrogen and the sample was stirred for an additional 7 days and dialyzed against PBS (molecular weight cut off 10,000 Da). The resulting fibrils were checked by EM and the purity was confirmed by the absence of oligomers using anti-oligomer antibody. The same protocol was used to prepare IAPP fibrils. Aβ and IAPP oligomer mimics were prepared as previously described [27] The synthesis of IAPP C-terminal thioester analog lacking cysteine residues (KANTATAATQRLANFLVHSSNNFGAILSSTNVGSNTY-SR), was also carried out according to the methods described [27]. The antigens were each used to immunize two New Zealand white rabbits (Pacific Immunology Corp., Ramona, CA, 92065) according to protocols approved by IACUC. Each rabbit immunized with 500 μl of antigen in complete Freund's adjuvant (CFA), and then boosted twice at four week intervals with 500 μl of antigen in Incomplete Freund's Adjuvant (IFA).

### Fibril and oligomer preparation

Aβ fibrils and fibrillar oligomers were prepared by dissolving 0.3 mg of lyophilized Aβ42 in 150 ul of hexafluoro-2-propanol (HFIP) for 10–20 minutes at room temperature. The resulting Aβ solution was added to DD H_2_O in a siliconized Eppendorf tube to 80 uM concentration. After 10–20 min incubation at room temperature, the samples were centrifuged for 15 min. at 14,000 × G and the supernatant fraction (pH 2.8–3.5) was transferred to a new siliconized tube and subjected to a gentle stream of N_2 _for 10 min to evaporate the HFIP. The sample was then stirred at 500 RPM using a Teflon coated micro stir bar for 24 hours at 22°C. This method was originally reported for preparing A11 positive prefibrillar oligomers [19], but more recent work indicates that it also produces fibrillar oligomers that are OC positive. Fibrils were separated from fibrillar Aβ42 oligomers by centrifuged at 100,000 × G for 1 hour at 4°C. The supernatant containing fibrillar oligomers and pellet fraction containing fibrils were separated and collected. The pellets were resuspended in an equal volume of H_2_O. Alternatively, 1 mg of lyophilized Aβ42 was dissolved in 200 μl of DMSO and incubated at room temperature for 10–15 minutes to form fibrillar oligomers. The fibrillar oligomers in DMSO were fractionated according to size using a TSK-GEL SuperSW2000 column (Tosoh Bioscience LLC) in 10 mM Phosphate, pH 7.4 at a flow rate of 0.3 ml/min.

Prefibrillar oligomers that are OC negative were prepared as previously described [22]. Aβ42 stock solutions (2 mM) were prepared by dissolving the lyophilized peptide in 100 mM NaOH followed by water bath sonication for 30 s. The oligomerization reaction was initiated by diluting the stock solution in phosphate buffered saline (PBS), pH = 7.4, 0.02% sodium azide (45 μM final Aβ_42 _concentration, final pH = 7.4) and incubated at room temperature for up to 15 days. Oligomer formation was monitored by dot blot with A11 and OC polyclonals.

ADDLs were prepared according to Lambert et al [23]. Aβ42 peptide was initially incubated in HFIP at room temperature for 1 hour. The HFIP was evaporated under a gentle stream of N_2_. The remaining Aβ42 was dissolved in anhydrous DMSO at 5 mM, diluted into cold phenol red-free F12 medium and aged at 4°C for 24 hours. The final peptide concentration was 80 μM.

Q36 fibrils were prepared by dissolving Q36 in 10 mM HEPES/100 mM NaCl at a concentration of 45 μM and incubating with stirring at 25 C for 6 days. Fibril formation was confirmed by EM and ThT. Q36 oligomers were prepared by dissolving Q36 in 1:1 (vol:vol) TFA:HFIP at 2 mM and diluting it to 45 μM in PBS and incubating with stirring for 6 days. Oligomer formation was confirmed with A11 antibody.

### ELISA, dot blot, Western blot assays and Immunohistochemistry

ELISA, dot blot and western blots assays were done as previously described [27]. Brain tissue from autopsy cases was provided by the University of California Alzheimer's Disease Research Center and the Institute for Brain Aging & Dementia Brain Tissue Resource. For single-labeling experiments, 50 μm 4% paraformaldehyde-fixed sections containing the hippocampus and entorhinal cortex or the midfrontal cortex from an AD case (Case #1 – 65 year old female, 7.4 hour post mortem interval, MMSE = 21 15 months prior to death with a Braak & Braak stage of VI) were washed with 0.1 M Tris-buffered saline (TBS), pH 7.5, and then pretreated with 3% hydrogen peroxide in 10% methanol to block endogenous peroxidase activity. Sections were subsequently washed in TBS with 0.1% Triton X-100 (TBS-A) and then blocked for thirty minutes in TBS-A with 3% bovine serum albumin (TBS-B). In a series of preliminary studies, the effects of different concentrations of formic acid during a pretreatment phase was determined to have little effect on the extent or intensity of OC labeling of fixed tissue (data not shown) and thus this step was eliminated from the protocol. Sections were incubated overnight at room temperature in OC at a dilution of 1:10,000. Following two washes with TBS-A and a wash in TBS-B, sections were incubated in either goat anti-mouse or goat anti-rabbit biotinylated anti-IgG and then in avidin biotin complex (ABC) (Vector Laboratories, Burlingame, CA, USA). Antibodies were visualized using 3,3'-diaminobenzidine (DAB, Vector Laboratories). For quantification experiments, the frontal cortex from all cases used for quantification was immunostained in single experiments to reduce variability in the image analysis procedures and all immunohistochemical procedures were identical for the OC antibody. To determine the specificity of the OC antibody, IgG purified serum at a concentration of 1:10,000 was preincubated in 10× and 100× concentration of OC peptide for 2 hours at RT. Subsequently, a section from the midfrontal cortex was incubated in the OC antibody/peptide solution and processed for immunohistochemistry. Sections were counterstained with cresyl violet.

### Mouse strain and tissue collection

Hemizygous human IAPP transgenic mice (FVB-tg(IAPP)6Jdm/-A^vy^/A) were characterized in details elsewhere [28]. For this study we used 24 wk old mice. Before collection of mouse pancreata, the heart was perfused with 10 ml of 4% paraformaldehyde. The pancreas was dissected in cold PBS, fat and lymph nodes trimmed, the pancreas weighed, fixed in 4% paraformaldehyde at 4°C for 24 h then frozen in OCT.

### Immunofluorescence and confocal microscopy

An additional AD case was used for confocal studies. Case #2 was a 95 year old female with a post mortem interval of 5.5 hours and a MMSE score of 12, 6.3 months prior to death. Sections containing the midfrontal cortex were incubated in OC overnight (1: 5,000) and positive labeling was detected using anti-rabbit IgG Alexa Fluor 568 (Molecular Probes, Eugene, OR; 1:200). Alexa Fluoro 488 (Molecular Probes, Eugene, OR; 1:200) was subsequently used to visualize LOC (1:5,000). The order of the primary antibodies was also reversed in additional experiments and the results were similar. Because both antibodies were raised in the same species (rabbit) an intervening formaldehyde treatment was used between the first and second immunolabel [29]. Sections were allowed to dry on slides prior to rehydration and coverslipping with VectaShield (Vector Laboratories, Burlingame, CA, USA). Confocal images were collected on an Olympus IX70 inverted microscope and a BioRad Radiance 2000 Laser Scanning System using a 40, 60 or 100× objective for image analysis. Each antibody label was excited and scanned using lambda strobing and barrier filters at 510 and 480 nm. A z-series scan at either 0.5 or 1 μm intervals was captured to determine the spatial colocalization characteristics of OC with LOC.

## Competing interests

CG and RK are paid consultants for Kinexis, Inc.

## Authors' contributions

RK prepared the OC, LOC and I11 antigens and antisera and did the initial chearcterization of their specificity. EH, FS, TS and CWC did the immunohistochemistry and immunofluorescence on human AD tissue. MN, LM, JW, LB and SR prepared prefibrillar and fibrillar oligomer samples and conducted the dot blot and western blot analysis of the samples. JT did the western blot analysis of human AD brain lysates. TG and PB conducted the Immunofluorescence analysis of IAPP Tg mouse pancreas. CG participated in concept, design, data analysis and manuscript preparation. All authors read and approved the final manuscript.
